# Study on Potential of Meridian Acupoints of Traditional Chinese Medicine

This article has been retracted.

**DOI:** 10.1155/2021/5599272

**Published:** 2021-03-03

**Authors:** Qiuping Li, Tianxia Zhao, Xin'an Wang, Changpei Qiu, Bing Zhou, Hu Wang, Bo Wang

**Affiliations:** The Key Laboratory of Integrated Microsystems, Peking University Shenzhen Graduate School, Shenzhen 518055, China

## Abstract

In recent years, Traditional Chinese Medicine (TCM) has attracted more and more attention due to its good therapeutic effect, low cost, and convenience. This research is also a part of the goal of the modernization of TCM. Based on the meridian electric potential acquisition system independently developed by our project team, in this paper, we designed the human body's meridian electric potential acquisition scheme. We use principal component analysis (PCA) to prove that the meridional potential signal is derived from the ECG signal. Then, Inception ResNet V2 was used to classify acupoints and nonacupoints. Finally, the classification accuracy rate reached 86.59045265, and the F1 score = 0.72161642. This shows that acupoints and nonacupoints can be distinguished by their surface potential.

## 1. Introduction

Meridian theory is a basic theory that expounds the concept of human body's meridian, the composition, circulation distribution, physiological function, pathogenesis changes, and the relationship between the meridian system and zang-fu organs, body officials and orifices, qi, and blood and is an important part of the theoretical system of Traditional Chinese Medicine. The meridian system is composed of meridians and collaterals. The meridians include the twelve meridians, the eight odd meridians the twelve tendons, and the twelve skin parts attached to the twelve meridians. The twelve meridians, which are the meridians to which the twelve zang-fu organs belong, are the core part of the meridians system, which is called Jing. There are relatively few quantitative studies of channels and collaterals in science.

In recent years, Traditional Chinese Medicine (TCM) has been gaining more and more attention as the traditional therapy of complementary and alternative medicine (CAM) in the world due to its simplicity, convenience, efficiency, and cheapness [1–3]. There is a growing amount of studies on specificities of meridian acupoints through biophysics [4–6], electrophysiology [7–9], infrared imaging [3, 10], and so forth.

In September 2015, the United Nations General Assembly accepted the 2030 Development Agenda, which has included 92 paragraphs, and Paragraph 91 defined 17 sustainable development goals (SDGs) and 169 associated targets [11]. Big data are widely recognized as being one of the most powerful drivers to promote productivity, improve efficiency, and support innovation. It is highly expected to explore the power of big data and turn big data into big values [12]. Effective energy efficiency and effective resource efficiency are to bring new views and potentials of green metrics for the future times of big data [13]. The world is witnessing an unprecedented growth of cyber-physical systems (CPS), which are foreseen to revolutionize our world via creating new services and applications in a variety of sectors such as environmental monitoring, mobile health systems, and intelligent transportation systems [14]. Combining big data with TCM will bring about important social value and economic benefit.

Acupoints distributed in the meridian system provide some unique ways of signal transmission and information processing, including electrical information [8]. However, up to now, there are few researches on the modeling of meridian system from the perspective of electronic information transmission. In addition, these studies mainly explored the hysteresis characteristics of meridian system through electronic acupoint stimulation signals [15] rather than directly exploring through acupoint electric potential signals [8, 10]. In some papers, the characteristics of parts of the body's meridians were studied [16–18], but rarely from the holistic theory of Chinese medicine, the systematic study of the twelve meridians was done in a human body. Based on the holistic view of Traditional Chinese Medicine, this study designed and realized the experimental study of human twelve meridians electric potential collection based on the multichannel human meridians electric potential collection system independently developed by the project team.

## 2. Acquisition System Structure

Previous studies on meridian acupoints failed to conduct a comprehensive collection experiment on the acupoints of the twelve meridians in the human body. In this paper, a multichannel and extensible human body meridian system electrical potential signal acquisition system, with characteristics of adjustability and scalability, has been designed. Improved input mode of electrodes decreases the contact area with skin. Detection circuits can change gain to suit different amplitudes of meridian electric potential signals. Modularizing analog circuits into a PCB board increases the degree of parallelism of the whole system. Software based on LabView is flexible to change the number of channels, sampling frequency, and range.

As shown in Figure 1, the structure of the whole system consists of two important parts, hardware and software. The former includes a group of electrodes, several detection boards, and an acquisition card. The latter is an acquisition system with a sampling controller and a database. The amplitude range of potential is from 0.05 to 20 mV, while the frequency range is from 5 to 500 Hz.  Figure 2 shows the circuit board of the multichannel acupoint potential acquisition system.

In this design, because of the advantages of Ag/AgCl electrode in cost and safety, the Ag/AgCl electrode is used. Each electrode is 2.5 centimeters in diameter. Each test plate has 7 electrodes: 5 test electrodes, 1 reference electrode, and 1 DRL electrode. The reference electrode connects the body to a common ground on the board to resist common-mode interference and reduce noise, while the DRL electrode achieves the same goal by rapidly discharging through a feedback loop. At the same time, the electric conductor is shielded to reduce the noise interference.

The acquisition card converts continuous analog voltage output by the detection board into discrete digital values and supports up to 64 channels of ADC with a total sampling rate of 250 K/s.

The main functions of the board multiplex detection circuit are amplification and filtering. After testing, acupoint electrical signals have the characteristics of small amplitude and low frequency. To take full advantage of the resolution of the ADC, the gain is adjustable so that the output voltage range of each channel is consistent with the supply voltage. On the other hand, if a high-gain single-stage amplifier is used, both external electromagnetic interference and the polarization voltage between the electrode and the skin may saturate the amplifier and lose useful information. This design adopts two-stage amplification, and appropriate signal filtering circuit is used between the two stages.

The electrode group is fitted and set on the body surface, and the electrical signal acquisition device on the body surface starts to supply power.

  Step 1. Initialize the body surface electrical signal acquisition device.
  Step 2. The multichannel detection circuit is used to obtain the human body surface electrical signal. If the human body surface electrical signal is not obtained, it is reinitialized. Otherwise, Step 3 is performed.
  Step 3. Set the channel of the detection circuit of the detection board.
  Step 4. Set the voltage range of the detection board.
  Step 5. Set the sampling rate of the acquisition card.
  Step 6. Judge whether the output waveform is correct and execute Step 7 correctly; otherwise, reinitialize.
  Step 7. Store the electrical signals of the human body surface converted into digital signals.
  Step 8. Judge whether all the samples have been completed. After the bits have been completed, reinitialize and continue to collect again.

Complete all samples and end the collection.

## 3. Meridian Potential Measuring Experiment

In the experiment, two groups of experiments were conducted for the collection of electrical signals in the twelve-meridian system of the human body. All channels in group *a* corresponded to acupoints on the meridians. Half of the channels in group *b* were used to monitor acupoints and half of the channels were used to monitor nonacupoints. Medical semicircular ECG electrodes were employed for the signal detection at measured acupoints. Additionally, the acupoints should be easy to measure so as to avoid the measuring deviation brought by undesirable conditions. While the left knee was regarded as a reference acupoint, the left elbow was used as the grounding point.  Figure 3 shows the experimental scene.

Ten healthy volunteers (five males and five females), aged 22 ± 3 years, were graduate students recruited from Peking University Shenzhen Graduate School. Ten stroke patients volunteers from Shenzhen Hospital of Traditional Chinese Medicine were 50 to 70 years old. All volunteers gave informed consent. The volunteers accepted the investigation and cooperated to complete the experiment. They have signed the information consent form. Each subject was measured only one hour after or before having foods or fierce sport. During the measuring procedure, the subject was required to keep quiet, turn off all the telecommunication devices, and take all metal items off the body.

Figures 4to 15 show the twelve meridians' points collected and the control acupoints. Group *a* is the selected meridian acupoints for testing. About half of the channels in group *b* were used to monitor nonacupoints. The numbered points identified in the figure are the nonacupoints to be monitored. Each set of potential acquisition experiments lasted 3 minutes.

## 4. Experiments and Results Analysis

### 4.1. Data Processing and Analysis

The first step is to remove power frequency interference, because the power frequency interference usually does not appear in the form of 50 Hz alone but often appears in the form of frequency multiplication multiple harmonics. Therefore, this data preprocessing is aimed at removing 50 Hz, 100 Hz, and 150 Hz. In the specific part of the algorithm, the Butterworth band-stop filter is used to remove the specified frequency signal, because the Butterworth filter is flat in the passband and has good linear phase characteristics, which can meet our requirements. The order of band-stop filter is 4. Because the band-stop filter can only filter out one frequency range but not a single frequency, a very small frequency range is adopted in this paper. Taking the signal of 50 Hz as an example, the algorithm is used to filter out the signal of 49 Hz–51 Hz, which also meets the requirements.  Figure 16 is the spectrum diagram of the signal before and after the removal of power frequency interference.

### 4.2. The Data of Cutting

In this experiment, 5-second data is used as a sample for data preprocessing. Since the sampling frequency of LabVIEW software platform is 1000 Hz, 7500-point data are classified as a sample. Since the experimental data collected are not strict three-minute data, the data of less than 7500 points is discarded in the end. The data of acupoint is labeled as 1, the data of nonacupoint is labeled as 0, and the final data is saved as NumPy data format for the convenience of subsequent algorithm invocation.

### 4.3. Classification Algorithm

The goal of our classification is to distinguish between acupoints and nonacupoints. The electrical potential signals collected at acupoints and nonacupoints on the meridian are labeled. The collected meridional potential signals were processed and found to have the characteristics of ECG signals as in Figure 17.

The extractor is based on Inception ResNet V2 with high performance in the current CV architecture [19]. It is characterized by parallel multisensory fields and can integrate multiscale features to better extract sample information [20]. It can adjust the gravity of data flow in each bypass and parallel multidimensional learning. Higher performance is traded for larger scale, which is not too burdensome for a one-dimensional ECG signal [21–23].

Minor modification is conducted to fit input length. In Inception ResNet V2, two continuous 3^*∗*^3 convolution layers are used to replace one 5^*∗*^5 convolution layer, which can reduce parameters while maintaining the inception field. Considering that this approach is invalid for one-dimensional samples, 1^*∗*^5 convolution layer is implemented as substitution.

### 4.4. Result

Two-thirds of the data are for training and one-third is for testing. The training accuracy of the test set is 86.59% and the F1 score is 0.7216. The results of model training are as follows: Figure 18 shows the training set's global loss function curve.  Figure 19 shows comparison of loss function between the training set and the test set.  Figure 20 shows the comparison of accuracy between the training set and the test set.  Figure 21 shows the F1 score of this classification model.

## 5. Discussion

The results show that the electrical potential signals detected in the body's meridians all have ECG characteristics.

To verify that the above signals are derived signals of ECG. 138 samples of ECG signals and 138 samples of acupoint electrical signals were taken for principal component analysis (PCA), respectively. Similarities and differences of data are classified and explored by using PCA [24–28]. The significance of PCA is to create small variables known as Principal Components (PCs) that work on the variance estimation theory. The covariance matrix explains the relationship between two signals:

(1) $$\begin{array}{c} s_{x}=\frac{1}{n-1}xx^{T}. \end{array}$$

The basic formula for covariance is expressed as

(2) $$\begin{array}{c} \mathrm{cov}\left(x,y\right)=\frac{\sum_{i=1}^{n}\left(x_{i}-\bar{x}\right)\left(y_{i}-\bar{y}\right)}{\left(n-1\right)}. \end{array}$$

Data of 1 second was taken from each sample. Since the sampling frequency was 1000 Hz, there were 1000 points of data in a sample. The 1000-point data can be regarded as 1000 feature points of a sample, and the final dimension *K* = 3 is set in the PCA algorithm to facilitate visualization. In other words, after PCA treatment, the dimensions of 1000 interrelated and related feature points are reduced to 3 independent points that can represent the sample features. Finally, the three feature points of each sample were set as *x*-, *y*-, and *z*-axes for three-dimensional scatter plots. The points of electrical signals at acupuncture points were set as red, and the points of ECG signals as blue. That is to say, there should be 138 red points and 138 blue points in the three-dimensional diagram. It can be seen that most of the points of the two colors in the figure are in the same region in Figure 22. This indicates that the electrical signals of the body's meridians are very similar to ECG signals. In other words, the acupoint potential signal is derived from the ECG signal.

## 6. Conclusion

Our study showed that the electric potential is detected along the meridians all over the body, and it is found that the electric potential signals have the characteristics of ECG signals, or the electric potential signals of the human meridians should be the derived signals of ECG signals. The results of this trial would help to prove that in Chinese medicine the heart controls mental activities theory. Then we tried to classify the acupoint and nonacupoint by the collected electric potential signals, and finally we got the classification accuracy rate of 86.59% and F1 score of 0.7216. It is indicated that acupoints and nonacupoints can be distinguished by their surface potential. In the following work, we will further analyze the potential characteristics of meridian acupoints. We will analyze the differences between the meridians and collaterals; meanwhile we will analyze the population with related diseases to evaluate the severity of the disease from the quantitative analysis of the meridian potential.

## Figures and Tables

**Figure 1:** The structure of the meridian electric potential acquisition system.

**Figure 2:** The circuit board of the multichannel acupoint potential acquisition system.

**Figure 3:** The experimental scene.

**Figure 4:** Lung meridian of Hand-Taiyin. 1a. Shaoshang-Yuji-Lieque-Chize-Tianfu-yunmen-Zhongfu. 1b. Shaoshang -②-Lieque - Chize -⑤ -Yunmen-⑦.

**Figure 5:** Hand Yanming large-intestine meridian. 2a. Shangyang -Hegu - Pianli - Quchi - Binao - Jianyu -Tianding. 2b. Shangyang -② - Pianli - Quchi -⑤ - ⑥ -Tianding.

**Figure 6:** Stomach meridian of Foot Yangming. 3a. Renying - Quepen - Futu -Liangqiu - Zusanli - Xiajuxu – Jiexi. 3b. Renying - ② - Futu -④ - Zusanli - ⑥-Jiexi.

**Figure 7:** Shaoyin Heart meridian of Hand. 4a. Shaofu – Shenmen –Lingdao – Shaohai – Qingling. 4b. Shaofu – Shenmen –③ – Shaohai – ⑤.

**Figure 8:** Spleen meridian of the Foot-Taiyin. 5a. Jimen-Xuehai-Yinlingquan -Diji -Sanyinjiao-Shangqiu- Gongsun. 5b. Jimen- ②-Yinlingquan -④-Sanyinjiao-⑥- Gongsun.

**Figure 9:** Sanjiao meridian of Hand-Shaoyang. 6a. Guanchong-Zhongzhu -Zhigou-Tianjing-Jianliao- Tianliao-Tianyou-Ermen. 6b. Guanchong-② -Zhigou-④-Jianliao-⑥-Tianyou-Ermen.

**Figure 10:** Foot-Taiyang bladder meridian. 7a. Dazhu -Fufen -Xinshu -Shenshu -Weizhong-Feiyang -Kunlun. 7b. ① -Fufen -Xinshu -④ -Weizhong-⑥ -Kunlun.

**Figure 11:** Hand Taiyang small-intestine meridian. 8a. Shaoze-Houxi-Yanglao -Zhizheng -Xiaohai -Jianzhen – Dazhui. 8b. Shaoze-Houxi- Yanglao -④ - Xiaohai -⑥-⑦.

**Figure 12:** Kidney meridian of Foot-Shaoyin. 9a. Shufu-Bulang -Youmen-Mangshu-Yingu (Yinlingquan)-Taixi - Shuiquan. 9b. Shufu -②Youmen-④-⑤-Taixi-Shuiquan.

**Figure 13:** Pericardial meridian of Hand-Jueyi. 10a. Zhongchong-laogong-Daling-Neiguan-Ximen-Quze – Tianquan -Tianchi. 10b. Zhongchong-②-Daling-④-Ximen-⑥-⑦ -tianchi.

**Figure 14:** Gallbladder meridian of Foot-Shaoyang. 11a. Qiuxu-Yangjiao-Yanglingquan-Zhongdu-Jingmen-Riyue-Jianjing-Yangbai. 12b. ①-Yangjiao-③-④-Jingmen-Riyue-⑦-Yangbai.

**Figure 15:** Liver meridian of Foot Jueyin. 12a. Dadun-Zhongfeng-Ligou-Xiguan-Ququan-Yinbao-Zhangmen-Qimen. 12b. Dadun-②-Ligou-④-⑤-Yinbao-⑦-Qimen.

**Figure 16:** (a) and (b) are the spectrum diagrams before and after power frequency interference is removed, respectively.

**Figure 17:** Electric potential diagram of meridian acupoints.

**Figure 18:** Training set's global loss function.

**Figure 19:** Comparison of loss function between the training set and the test set.

**Figure 20:** Comparison of accuracy between the training set and the test set.

**Figure 21:** The F1 score of this classification model.

**Figure 22:** Three-dimensional diagram of PCA results of meridional potential signal (the red points represent the electric potential signals at meridian acupoints, and the green ones represent the standard ECG signals).

## Data Availability

The data that support the findings of this study are available from the corresponding author upon reasonable request. In addition, since the data involves personal privacy issues, it is necessary to contact the corresponding author and relevant parties to sign the data confidentiality agreement.
